# Neural Network-Based Study about Correlation Model between TCM Constitution and Physical Examination Indexes Based on 950 Physical Examinees

**DOI:** 10.1155/2020/8812678

**Published:** 2020-09-01

**Authors:** Yue Luo, Bing Lin, Shuting Zhao, Li He, Chuanbiao Wen

**Affiliations:** ^1^Chengdu University of Traditional Chinese Medicine, No. 1166 Liutai Avenue, Wenjiang District, Chengdu 611137, China; ^2^Affiliated Hospital of Chengdu University of Traditional Chinese Medicine, No. 37 Shierqiao Avenue, Jinniu District, Chengdu 610075, China

## Abstract

**Purpose:**

To establish the correlation model between Traditional Chinese Medicine (TCM) constitution and physical examination indexes by backpropagation neural network (BPNN) technology. A new method for the identification of TCM constitution in clinics is proposed, which is trying to solve the problem like shortage of TCM doctor, complicated process, low efficiency, and unfavorable application in the current TCM constitution identification methods.

**Methods:**

The corresponding effective samples were formed by sorting out and classifying the original data which were collected from physical examination indexes and TCM constitution types of 950 physical examinees, who were examined at the affiliated hospital of Chengdu University of TCM. The BPNN algorithm was implemented using the C# programming language and Google's AI library. Then, the training group and the test (validation) group of the effective samples were, respectively, input into the algorithm, to complete the construction and validation of the target model.

**Results:**

For all the correlation models built in this paper, the accuracy of the training group and the test group of entire physical examination indexes-constitutional-type network model, respectively, was 88% and 53%, and the error was 0.001. For the other network models, the accuracy of the learning group and the test group and error, respectively, was as follows: liver function (31%, 42%, and 11.7), renal function (41%, 38%, and 6.7), blood routine (56%, 42%, and 2.4), and urine routine (60%, 40%, and 2.6).

**Conclusions:**

The more the physical examination indexes are used in training, the more accurate the network model is established to predict TCM constitution. The sample data used in this paper showed that there was a relatively strong correlation between TCM constitution and physical examination indexes. Construction of the correlation model between physical examination indexes and TCM constitution is a kind of study for the integration of Chinese and Western medicine, which provides a new approach for the identification of TCM constitution, and it may be expected to avoid the existing problem of TCM constitution identification at present.

## 1. Introduction

In the Traditional Chinese Medicine (TCM) concepts, a person's constitution refers to such inherent qualities that are comprehensive and relatively stable in the morphological structure, physiological functions, and psychological states, which are formed during one's life on the basis of natural endowment and postnatal maintenance, which are personal features adapting to natural and social environment formed in the growth and development process of human [1, 2]. Numerous classics of TCM explain the theories of TCM constitution. It is recorded that “people here are living the same life, with the same age and the same clothes. When a strong gale or rainstorm attacks, some fall ill, some not; or everybody gets ill or nobody gets ill at all. What is the reason for this? It is because a person with fragile physique cannot survive the deficient winds in the four seasons, while a person with strong physique can easily get by” [3] in *The Inner Canon of Huangdi*, a classic work as the theoretical basis guiding TCM. This paragraph underlines the dominant role a person's constitution plays during the onset of illness. In another work by Wang, who is the founder of the TCM Constitution and master of Chinese medicine, the *Theory of TCM Constitution*, which summarizes and extends the TCM constitution, it is proposed that lots of factors can influence a human's constitution such as natural factors, age, gender, spirit, diet, living condition, and geographic environment. [1]. According to the basic theory of TCM and clinical survey, Wang also proposed the classification of nine kinds of TCM constitution, which are peaceful type, qi-deficient type (qi is the vital energy that runs through a human body), yang-deficient type (yang refers to the heat and energy that a human body possesses), yin-deficient type (yin is the opposite of yang, referring to the body fluid that cools and quiets a body), phlegm-damp type, damp and hot type, blood stasis type, qi depression type, and special type [4]. TCM theory believes that an individual's special constitution can cause him/her to be particularly sensitive to some diseases, and such particularity of an individual's constitution will directly affect the onset and progress of a disease [5]. Therefore, it is necessary for disease preventive treatment to prevent disease onset and exacerbation by distinguishing constitution.

Figure 1 shows the neural network model of physical examination indexes and TCM constitutional types. The input of backpropagation neural network (BPNN) is physical examination indexes, and the output is TCM constitution types. *X*_1_, *X*_2_,…, *X*_n_ refers to the quantified and normalized physical examination indexes; Y_1_, Y_2_,…, *Y*_m_ refers to the calculated outputs by the BPNN, corresponding to the TCM constitution types; W refers to weights from the input layer to hidden layer, and V refers to weights from the hidden layer to output layer.

Nowadays, human can live longer than before. However, stress from job and life is increasing, which causes many people to fall ill [6]. Physical examination is becoming an important approach to diagnose and prevent diseases. Physical examination indexes are the quantitative indexes used by Western medicine, which employ multiple physical and chemical parameters such as blood routine indexes, urine routine indexes, liver function indexes, and renal function indexes, to indicate physical conditions of a person. In the field of TCM, identification of constitution is the basis for formulating individualized preventive and health care measures, and it is also the prerequisite for getting rid of subhealth status and realizing “treatment without disease” [7, 8]. The current TCM constitution identification methods include TCM doctors' artificial identification, gene classifier, meridian thermal sensitivity measurement, pulse wave frequency-domain analysis, and scale method. All the methods above have been proved to have some problems: (1) the artificial identification of TCM doctors is susceptible to the doctor's theoretical level and clinical experience and faces the shortage of TCM doctors, which cannot meet the needs of constitutional identification. (2) The cost and technical requirements of genetic classification, meridian thermal sensitivity measurement, pulse wave frequency-domain analysis, and other identification methods are high. Some are still in the exploration stage. So it is not conducive to popularization and application [9, 10]. (3) The scale method, organized to form and administered by the State Administration of TCM of the People's Republic of China, is compiled by the China Association of Chinese Medicine Constitution Branch. In 2009, the document “Traditional Classification and Judging Standards for TCM Constitution,” which guides and regulates the research and application of TCM constitution, was published [11]. Although the scale method has been widely used, some experts have proposed that the scale has the problems of the abolishment of observation, auscultation and olfaction, and palpation and pulse feeling in the TCM constitution identification, which are called “the diagnosis of Wang, Wen, and Qie” in Chinese medicine and the loss of the overall concept of Chinese medicine [12–15]. Therefore, parts of hospitals actually carry out the constitution identification by combining the scale method with the three clinical diagnosis methods of TCM. In this situation, the process of TCM constitution identification goes through two stages, from the independent diagnosis to the comprehensive analysis, which has the problems of complicated process and low efficiency. At the same time, the scale is susceptible to subjective factors of the tester [16]. Thus, it is quite necessary to explore a new TCM constitution identification method.

In this situation, it proposes the research based on the integrative between Chinese and Western medicine, for which it uses BP artificial intelligence neural network (BPNN) technology and the samples from clinical of hospital to establish the network model of physical examination indexes and TCM constitution. In the correlation network model, the TCM constitution is quantitatively analyzed by physical examination indexes. It provides a new approach for the identification of TCM constitution, and it may be expected to avoid the existing problem of TCM constitution identification at present.

The remainder is organized as follows.  Section 2 reviews research efforts on correlation between TCM constitution and physical examination indexes and identification of TCM constitution.  Section 3 describes the study method on building the correlation model. In Section 4, the proposed model for TCM constitution and physical examination is assessed in multiple clinic experiments, and various numerical results are presented and discussed. Finally, Section 5 concludes and discusses future extensions.

## 2. Related Work

There were some recent researches about the correlation between TCM constitution and physical examination indexes. For example, Deng and Lu made combined analysis over physical examination indexes and constitutional types through clinical study and application, aiming to provide better regulation solutions for patients [17–20]. Using physical examination indexes and constitutional types of 331 community elderly, Ren and Li from Beijing Shijingshan District TCM Hospital performed a correlation analytical study, from which some conclusions that can guide clinical practice are drawn [21]. There are some other correlation researches, such as combined analysis over TCM constitution and physical examination indexes through different diseases like obesity, cerebral apoplexy, and hypertension. With statistical or regression analysis, they made the similar conclusions that some constitution types correlated with physical examination indexes were associated with a certain disease [22–32]. All the above studies show that there is a certain correlation between physical examination indexes and TCM constitution. But they only focused on the correlation between some physical examination indexes and some physical constitution types by using traditional methods of data statistics and analysis. The above research is not only lacking in the overall situation but also has not provided a template for the correlation between physical examination indexes and TCM constitution.

In view of the problems existing in TCM constitution identification methods, there were also some studies on identification of TCM constitution in an automatic way. Zhang et al. proposed the design and implementation of an identification system for TCM constitution, which implemented the electronic questionnaire of identification for TCM constitution [33–36]. This method is based on the scale method mentioned above. In practice, one's constitution type is identification combining the result of the system and the result from TCM doctors' artificial identification, which causes the low efficiency. Liang proposed an automatic identification system of TCM constitution based on facial image features. According to the result of facial diagnosis, which is done by the system with digital image processing technology, TCM constitution can be distinguished automatically. However, the accuracy of the result is not high. Meanwhile, the study selected fewer facial features, and the selected features did not fully represent a person's constitution type [37]. Hong et al. proposed an approach for identification of TCM constitution based on the tongue manifestation [38]. Yet it depended on tongue diagnosis combining with questionnaire analysis, which is still in exploration. Bai proposed a way to distinguish TCM constitution based on BPNN [39]. For this approach, the TCM constitution was identified by combining inspection, inquiry, and palpation, which was more objective and intelligent. But the accuracy still needs to be enhanced, and its practicability remains to be verified. Xie proposed the realization of a platform for the identification of TCM constitution and data analysis, by which it could complete TCM constitution identification based on scale and tongue diagnosis and provide the function of data analysis. However, the analysis algorithm adopted in this study will lead to the platform speed being too slow. The tongue diagnosis analysis algorithm cannot accurately analyze the tongue image, and the accuracy of TCM constitution identification remains to be questioned [40].

The previous studies are short for efficiency, accuracy, and correlation template. As above, it is expected to provide a new approach for TCM constitution identification by considering the correlation between TCM constitution and physical examination indexes with overall view and constructing a correlation model. With the rapid development of artificial intelligence and machine learning technology, it is a new trend to employ machine learning and neural network in TCM for automatic and smart identification of TCM constitution. Products such as smart medical equipment, intelligent diagnosis and treatment, and intelligent image recognition, which have achieved rapid development, have been successfully applied in various fields. So, in this paper, it explored the approach with BPNN, to implement the identification of TCM constitution and to build the correlation model between TCM constitution and physical examination indexes from 950 physical examinees. The data about physical examination indexes and TCM constitutional types of the physical examinees were first collected and sorted out. The physical examination indexes were classified into four categories, namely, blood routine indexes, urine routine indexes, liver function indexes, and renal function indexes. These four categories of indexes combined with the corresponding TCM constitutional types of physical examinees were the original sample data. The effective data, obtained from proper organization of the original data, were initially divided into the training group data and test group data. Furthermore, the training group data were input into the BPNN, which was trained to establish physical examination indexes-TCM constitution-type network model. Finally, the test group data were input to verify the accuracy of the established neural network model. After the verified experiment, the accuracy of the training group and the test group was up to 88% and 53%, respectively, and the error was close to 0.001. Therefore, this research provides an automatic model to correlate physical examination indexes and TCM constitutional types, so as to use quantitative indexes of Western medicine to realize automatic and smart identification of TCM constitution and to provide a new way for TCM constitution identification.

The comparison between the previous studies and methods and the proposed method for constitution identification of TCM is shown in Figure 2.

The key contributions of this paper are summarized below:

1. A new approach to studying the correlation between TCM constitution and physical examination indexes is firstly proposed. BPNN algorithm is applied to build the correlation model, in which physical examination indexes are the inputs, TCM constitution types are the outputs, and Sigmoid function is the activation function. Then, it comprehensively analyzes the correlation of the two mentioned before and provides an automated relevance template.
2. A new method for identifying TCM constitution is proposed. It is successfully to construct a correlation model between physical examination indexes and TCM constitution. The model is verified by experiment with high accuracy and low error. It provides a smarter and more automatic way to realize the identification of TCM constitution types compared to the current ways including doctor and questionnaire.

## 3. Study Method

Neural network is a large-scale parallel distributed processor composed of simple processing units, which has characteristics in storing experiential knowledge and availability. It is similar in two ways to human's brain [41]:

1. Neural network acquires knowledge by learning from external environment.
2. The strength of interconnection neurons, the synaptic weight, is used to store acquired knowledge.

BPNN algorithm is a kind of artificial neural network technology that is intuitive, easily understood, and widely studied and used, with a powerful ability of nonlinear mapping and self-learning [42, 43]. It is also a kind of multilayered neural network that can be trained to learn the appropriate internal representations to allow learning any arbitrary mapping from input to output. A typical BPNN consists of three layers, i.e., input, hidden, and output layers, which are closely connected to each other [44].

The learning process of BPNN is composed of forward propagation and backpropagation. In the forward propagation process, the result is transmitted to the output layer after the data from the input layer are processed by neurons of hidden layer. The states of neurons in each layer only influence the state of neurons in the next layer. The process of backpropagation is started, while the computational output is not equal to the expected output. In the backpropagation process, error signal from an output layer is propagated up to an input layer via the hidden layer, and the link weight and offset are adjusted throughout the way. This process is finished until the accuracy reaches the requirement of algorithm. In fact, the BPNN algorithm aims at calculating a minimum error function. By repeated training of multiple samples, BPNN adjusts weight in a negative gradient of error function till the error converges to the least [45].

Based on the above theories, we adopted BPNN to establish the correlation model between TCM constitutional types and physical examination indexes in this work.

The effective data were sorted out from original data collected from the subjects, and 80% of which was input as training group data into the BPNN to establish the model. The physical examination indexes in the test group data, accounting for 20% of the effective data, were input into the network model to predict the corresponding TCM constitutional types. The reason for such percentage allocation will be discussed later. The effective data, which were randomly divided into the training group and the test group, covered the nine constitutional types of TCM as mentioned before.

### 3.1. TCM Constitutional Types-Physical Examination Indexes: BPNN Correlation Model Algorithm

The BPNN model for correlation between TCM constitutional types and physical examination indexes is shown in Figure 3. The detailed description of the algorithm is as follows.

In this model, it took physical examination indexes as input and TCM constitution types as output. The weight from the input layer to hidden layer was denoted as *ω*_*ij*_ and that from the hidden layer to output layer was denoted as *ω*_*jk*_; the offset from the input layer to hidden layer was denoted as *a*_*j*_, and that from the hidden layer to output layer was denoted as *b*_*k*_. The learning rate was *ç*. The excitation function was *g*_(*x*)_[46]. This study chose Sigmoid function (S-function) as the excitation function to establish the correlation model and to realize conversion of variable data and weight. Because S-function is nonlinear, its parameter values need to be in [0, 1], and the physical examination index can easily satisfy this condition. The equation of S-function is shown as follows:

(1) $$\begin{array}{c} g_{\left(x\right)}=\frac{1}{1+e^{-x}}. \end{array}$$

The training process of the algorithm is as follows:

1. Take random algorithm to initialize the weights *ω*_*ij*_ and *ω*_*jk*_ and the offset*a*_*j*_ and *b*_*k*_
2. According to formula (2), the BPNN algorithm calculates the hidden layer output *H*_*j*_ after inputting the quantitative physical examination indexes *X*_*i*_ of training group of sample
3. Employ formula (3) to calculate the predicted output *O*_*k*_, which represents the TCM constitution types
4. Compare the actual TCM constitution type quantified in the sample with the predicted value of the algorithm *O*_*k*_ and then employ equation (4) to calculate the error
5. The convergence of algorithm is judged according to the iteration number, the number of training group for the same batch and the error
6. If the convergence is achieved, stop to learn, which indicates the model is built
7. If it does not converge, reverse the revision weights *ω*_*ij*_ and *ω*_*jk*_ and the offset *a*_*j*_ and *b*_*k*_ while continue to train about the sample

After the model is built, the test (validation) process of the algorithm is as follows:

1. Input the physical examination indexes of test (validation) group
2. Calculate the hidden layer *H*_*j*_ and the output layer *O*_*k*_ based on the revised weights and offsets in the training process
3. Calculate the accuracy by comparing the output *O*_*k*_ of the model with the actual TCM constitution type quantified by the test group
4. Calculate the error
5. *O*_*k*_ is the predictive value of the correlation model

For the new data of the validation group, if the algorithm does not converge, the algorithm continues to reverse the revision weight and offset until the algorithm converges.

#### 3.1.1. Input Layer

Physical examination indexes, namely, blood routine indexes, urine routine indexes, liver function indexes, and renal function indexes, were used as input nodes of the network model.

#### 3.1.2. Hidden Layer

The number of hidden layer nodes, which was indicated as *n* in equation (2), was assigned from 1 to 10, respectively, to verify the accuracy and time efficiency of the algorithm. The hidden layer output was denoted as*H*_j_, which was calculated as follows:

(2) $$\begin{array}{c} H_{j}=g\left(\sum_{i=1}^{n}w_{ij}x_{i}+a_{j}\right). \end{array}$$

Neither too few nor too large number of hidden layer nodes can get a good convergence of the BP algorithm. Verification showed that when the number of hidden layer nodes was 5, both the convergence and time efficiency of the algorithm were satisfactory; therefore, in this paper, *n* = 5.

#### 3.1.3. Output Layer

The nine constitutional types were used as input nodes. The output layer output was denoted as *O*_*k*_, which was calculated as follows:

(3) $$\begin{array}{c} O_{k}=\sum_{j=1}^{n}H_{j}\omega_{jk}+b_{k}. \end{array}$$

In equation (3), *n* was the number of hidden layer nodes.

#### 3.1.4. Calculation of Error Δ

The error function was calculated as follows:

(4) $$\begin{array}{c} \Delta =\frac{1}{2}\sum_{k=1}^{m}{\left(Y_{k}-O_{k}\right)}^{2}, \end{array}$$

where *m* referred to the number of output layer nodes, *m* = 9. *Y*_*k*_ was the expected output (i.e., actual results of samples).

#### 3.1.5. Initialization and Updating of Weight

Random function was employed to generate a random value to initialize the weight. The equations for updating weight were as follows.

Weight from the input layer to hidden layer was

(5) $$\begin{array}{c} w_{ij}=w_{ij}+\eta H_{j}\left(1-H_{j}\right)x_{i}\sum_{k=1}^{m}\omega_{jk}\left(Y_{k}-O_{k}\right). \end{array}$$

And weight from the hidden layer to output layer was

(6) $$\begin{array}{c} \omega_{jk}=\omega_{jk}+\eta H_{j}\left(Y_{k}-O_{k}\right). \end{array}$$

#### 3.1.6. Initialization and Updating of Offset

Random function was employed to generate a random value to initialize the offset. The equations for updating offset from the input layer to hidden layer and from the hidden layer to output layer were

(7) $$\begin{array}{c} b_{k}=b_{k}+\eta \left(Y_{k}-O_{k}\right), \end{array}$$

(8) $$\begin{array}{c} a_{j}=a_{j}+\eta H_{j}\left(1-H_{j}\right)\sum_{k=1}^{m}\omega_{jk}\left(Y_{k}-O_{k}\right). \end{array}$$

### 3.2. BPNN Algorithm Flow

The neural network algorithm flow for correlation model of TCM constitutional types and physical examination indexes was as follows [26]:

1. Input the physical examination indexes of samples of training group.
2. Perform normalization of input data.
3. Initialize weight, offset, and learning rate.
4. Employ equation (2) to calculate hidden layer output.
5. Employ equation (3) to calculate output layer output.
6. Input TCM constitutional type data of samples.
7. Employ equation (4) to calculate error.
8. Employ equations (5)–(8) to update the weight and offset from the input layer to hidden layer and from hidden layer to output layer, respectively.
9. Judge whether convergence is achieved, i.e., whether the error reaches designated value; if convergence is achieved, proceed to next step; otherwise, return to step 4. Convergence of the algorithm indicates that the correlation network model of TCM constitutional types and physical examination indexes has been formed.
10. Input the physical examination indexes of the test group into the above established neural network model.
11. Predict the TCM constitutional types of test group.
12. Compare the prediction results of network model and the actual results of test group; calculate and output the final accuracy and error.

With the input of physical examination indexes, the type of TCM constitution can be automatically judged by the correlation model.

The above procedure flow is summarized in Figure 4.

### 3.3. Quantification and Normalization of Sample

According to physical examination index criteria adopted by health management center of the affiliated hospital of Chengdu University of TCM, the indexes in this paper were chosen as follows:

1. Blood routine indexes: 20 indexes including white blood cell and neutrophil cell population, lymphocyte population, monocyte, eosinophilia granulocyte, alkaline granulocyte, and percentage of neutrophil cell.
2. Urine routine indexes: 20 indexes including pH value, urine specific gravity, white blood cell, and red blood cell.
3. Liver function indexes: 11 indexes including total protein, albumin, and globulin.
4. Renal function indexes: 5 indexes including urea nitrogen, creatinine, trioxypurine, glucose, and carbon dioxide combining power.
5. All indexes of physical examinees: 56 indexes including blood routine index, urine routine index, and liver function index and renal function index.

Prior to applying TCM constitutional type data to neural network algorithm, the TCM constitutional types should be standardized. Taking into account the characteristics of neural network algorithm and activation functions, the TCM constitutional types were digitized and standardized. Conversion standards are shown in Table 1.

The physical examination indexes were also normalized by the custom algorithm which was not depicted owing to its simplicity. As the Sigmoid activation function discussed above is valued within [0, 1], the physical examination indexes have to be normalized so that the values are within [0, 1].

## 4. Experiments and Results

### 4.1. Data Collection

The 950 physical examinees, accepted by the health management center of the affiliated hospital of Chengdu University of TCM from January 2016 to March 2017, were used as study objects. Due to the security and confidentiality of the data, it took about 7–8 months to manually collect data, to entry data, and sort out data. The collected original data were cleaned, classified, and organized to form the effective data. The effective data were randomly divided into the training group and test group. In the experiment, the accuracy and error of the network model were verified using four different data size ratios of training over testing, i.e., 95%:5%,80%:20%, 60%:40%, and 50%:50%, respectively. The results indicated that when training group data: test group data = 80%:20%, the network model has the highest accuracy and the lowest error. Therefore, this study applied this percentage allocation to establish and verify the network model.

Blood routine indexes of 383 physical examinees, urine routine indexes of 186 physical examinees, liver function indexes of 564 physical examinees, renal function indexes of 313 physical examinees, and entire physical examination indexes of 133 physical examinees, as well as those physical examinees' corresponding TCM constitutional types, were used as effective data. 80% of the effective data was regarded as training data, while 20% was regarded as the testing data. All the samples, training group, and test group data covered the nine TCM constitutional types. For example, in the data samples of blood routine indexes, the distribution of TCM constitutional types is as shown in Figure 5.

As shown in Figure 4, it has a small number of special types, which are caused by a small number of people of these types in the world.

### 4.2. Algorithm Implementation

Visual Studio was employed to implement the neural network algorithm for the correlation between TCM constitutional types and physical examination indexes. Google's AI library and C# programming language were utilized for algorithm implementation. The number of iterations was set to 5000000; the accuracy and error were output once for every 1000 iterations (Algorithm 1).

### 4.3. Accuracy and Error Results

Accuracy and error are essential to verify the prediction data of a network model. The algorithm in this paper employed the blood routine examination, urine routine examination, liver function index, renal function index, and entire physical examination index data of training group to establish the neural network model and then used the test group data for model verification. The accuracy represents the ratio of the model prediction results to the actual results of the sample, and the error is calculated by the BP neural network algorithm, as shown in equation (4). If the accuracy is higher and the error is lower, the similarity between the predicted results of the model and the true clinical results is higher, which indicates that the model has a higher availability. Running time represents the time it takes to run the algorithm for every 1000 iterations of sample.

In order to construct and verify the correlation model between different physical examination indexes and constitution of TCM, we carried out, respectively, experiments for entire physical examination indexes, blood routine indexes, urine routine indexes, liver function indexes, renal function indexes, and corresponding constitution types of TCM and built the corresponding correlation model. The accuracy, error, and running time of every correlation model are shown in Table 2.

From Table 2, the following could be obtained:

  The training group and test group of liver function indexes-TCM constitution have an accuracy of 31% and 42%, respectively, and the error is 11.7.
  The training group and test group of renal function indexes-TCM constitution have an accuracy of 41% and 38%, respectively, and the error is 6.7.
  The training group and test group of blood routine indexes-TCM constitution have an accuracy of 56% and 42%, respectively, and the error is 2.4.
  The training group and test group of urine routine indexes-TCM constitution have an accuracy of 60% and 40%, respectively, and the error is 2.6.
  The training group and test group of entire physical examination indexes-TCM constitution have an accuracy of 88% and 53%, respectively, and the error is 0.001.

It is concluded that the more the physical examination indexes are, the more accurate the correlation model is, and the lower the error is.

In Figures 6 and 7, the horizontal axis of 1–5, respectively, represents the entire physical examination indexes-TCM constitution model, blood routine indexes-TCM constitution model, urine routine indexes-TCM constitution model, liver function indexes-TCM constitution model, and renal function indexes-TCM constitution model.

Figures 6 and 7 show that the accuracy is the highest of the entire physical examination indexes-TCM constitutional model.

Figure 8 illustrates the accuracy distribution in the training group of entire physical examination indexes-constitutional-type neural network model; the accuracy reaches 88% when the number of iterations is 1834000, and it goes stable while the number of iterations reaches 3481000.

Figure 9 illustrates the accuracy distribution in the test group of entire physical examination indexes-constitutional-type neural network model; the accuracy reaches 53% when the number of iterations is 171000, and it goes stable at the same time.

Figure 10 shows the error (the computational method is shown in equation (2)) distribution of entire physical examination indexes-constitutional-type neural network model. It points out that the error is less than 1 when the number of iterations reaches 81000 although it is high at the beginning.

Figure 11 illustrates the error distribution under 1. It depicts that the error decreases in a stable way, while the number of iterations reaches 3357000. It proves that the algorithm reaches convergent.

The above results prove that there is a relatively strong correlation between TCM constitution and physical examination indexes for the high accuracy and low error. It may reach the higher accuracy and lower error if the number of data increases.

## 5. Conclusions

In this paper, modern computer technology and AI neural network technology were employed to establish network models for physical examination indexes and TCM constitutional types. The data in the training group were used to establish the physical examination index-TCM constitution neural network model. And the data in the test group were used to verify the model. The results indicate that the more the physical examination indexes are, the more accurate the model is, and the lower the error is. For the entire physical examination indexes-TCM constitution correlation model, the training group and test group have an accuracy of 88% and 53%, respectively, and the error is 0.001. This value is higher than other experimental groups performed in this study such as urine routine examination indexes-TCM constitution model and liver function examination indexes-TCM constitution model. Verified by the text group data, this study shows that there is a relatively strong correlation between modern physical examination indexes and TCM constitutional types.

This paper fills the gaps about the researching of correlation between TCM constitution and physical examination indexes and provides the possibility for identification of TCM constitution based on the correlation model. The combined study of physical examination indexes and TCM constitution has profound meaning in exploring correlation between TCM and Western medicine, which would provide an associated automation template for both, in promoting TCM modernization and automatic and objective identification of TCM constitution in an innovative approach, which would be expected to avoid the problems existing in the current TCM constitution identification methods and in boosting preventive treatment of disease.

This paper uses clinical data and BP neural network technology which is widely used and matures in the field of artificial intelligence, to complete the construction of the physical examination indexes-TCM constitution network model, but this work still needs to be improved. For the volume of sample is not large enough, the future plans include improving algorithm and enhancing size of sample data, such as applying the remaining physical examination indexes, like the basic data of physical examination, blood lipid index, and the full set of transfusion index, and the corresponding TCM constitution, which are helpful to get a prediction model with high accuracy and low error, to do more experiments. In addition, the future endeavors will focus on identification of TCM constitution based on the correlation model. For example, the research will develop a system for identification of TCM constitution based on the correlation model. Then, the system will be applied in the identification of clinical TCM constitution to promote a new method of TCM constitution identification.

## Figures and Tables

**Figure 1:** Neural network model of TCM constitutional types and physical examination indexes.

**Figure 2:** The comparison between the previous studies and methods and the proposed method.

**Figure 3:** Neural network model of TCM constitutional types and physical examination indexes.

**Figure 4:** Neural network algorithm implementation procedures for physical examination indexes and TCM constitutional types.

**Figure 5:** Blood routine indexes-effective data of the training and test groups.

**Figure 6:** The accuracy chart of the learning group of different physical examination indexes-TCM constitutional model.

**Figure 7:** The correct rate chart of the test group of different physical examination indexes-TCM constitutional model.

**Figure 8:** Accuracy of the training group of entire physical examination indexes-constitutional type network model.

**Figure 9:** Accuracy of the test group of entire physical examination indexes-constitutional type network model.

**Figure 10:** Error of entire physical examination indexes-constitutional-type network model.

**Figure 11:** Error of entire physical examination indexes-constitutional-type network model (error<1).

**Algorithm 1:** Portions of code for building the correlation model.

**Table 1:** Standardization of TCM constitutional types.

SN	Constitutional type	Digitization representation
1	Peaceful type	0.1
2	*qi*-deficient type	0.2
3	*yang*-deficient type	0.3
4	*yin*-deficient type	0.4
5	Phlegm-damp type	0.5
6	Damp and hot type	0.6
7	Blood stasis type	0.7
8	*qi* depression type	0.8
9	Special type	0.9

**Table 2:** Accuracy results for different physical examination indexes, TCM constitution neural network models.

Name of neural network model	Accuracy of training group (%)	Accuracy of test group (%)	Error	Running time (time for every 1000 times iteration, sec)
Entire physical examination indexes-constitutional type	88 (top), 56 (stable)	53	0.001	0.1
Urine routine-constitutional type	60	40	2.6	0.051
Blood routine-constitutional type	56	42	2.4	0.063
Renal function-constitutional type	41	38	6.7	0.079
Liver function-constitutional type	31	42	11.7	0.063

## Data Availability

The 950 physical examinees, accepted by the Health Management Center of the Affiliated Hospital of Chengdu University of TCM from January 2016 to March 2017, were used as study objects.
